The article "Icariin Regulates the hsa_circ_0003159/eIF4A3/bcl-2 Axis to Promote Gastric Cancer Cell Apoptosis" was published in 2022. Journal: Evid Based Complement Alternat Med.

# Icariin Regulates the hsa_circ_0003159/eIF4A3/bcl-2 Axis to Promote Gastric Cancer Cell Apoptosis

**DOI:** 10.1155/2022/1955101

**Published:** 2022-07-15

**Authors:** Yanfen Yin, Wenwen Xu, Yanan Song, Zhou Zhou, Xin Sun, Fengli Zhang

**Affiliations:** ^1^Department of Oncology, The First Affiliated Hospital of Anhui University of Traditional Chinese Medicine, Hefei 230031, Anhui, China; ^2^The Graduate School, Anhui University of Traditional Chinese Medicine, Hefei 230038, Anhui, China; ^3^Department of Traditional Chinese and Western Oncology, The First Affiliated Hospital of Anhui Medical University, No. 120 Wanshui Road, High-tech Zone, Hefei 230088, Anhui, China

## Abstract

**Objective:**

To clarify the mechanism of icariin (ICA) promoting gastric cancer (GC) cell apoptosis by regulating circ_0003159/eIF4A3/bcl-2 axis.

**Methods:**

The mRNA or protein levels were detected by qRT-PCR or the western blot. The interaction between eIF4A3 protein and circ_0003159 or eIF4A3 protein and bcl-2 mRNA were validated by RNA pull down assays and the RNA immunoprecipitation (RIP) assay. The cell viability was measured by the cell counting kit (CCK)-8 kit. The cell apoptosis was measured by flow cytometry.

**Results:**

Compared with the group Vector, the ratio of cytoplasmic eIF4A3/nuclear eIF4A3 in the cell with circ_0003159 overexpression was significantly higher. RIP and RNA pull down results proved the interaction between eIF4A3 and circ_0003159. The RIP assay further validated the interaction between eIF4A3 and bcl-2. By gain or loss of the functional experiment, hsa_circ_0003159 was proved to recruit eIF4A3 to inhibit bcl-2 expression. Hsa_circ_0003159 regulates eIF4A3/bcl-2 to reduce GC cell viability and increase apoptosis Furthermore, ICA regulates hsa_circ_0003159/eIF4A3/bcl-2 axis to inhibit GC cell activity and induce GC cell apoptosis *in vitro*.

**Conclusion:**

These data showed that ICA could effectively reduce the GC cell activity and induce GC cell apoptosis via hsa_circ_0003159/eIF4A3/bcl-2 axis, which provides new theoretical evidence for the treatment of GC by ICA.

## 1. Introduction

Gastric cancer (GC) is a common malignant tumor of the digestive tract. China is one of the high incidence areas of GC, with 400 thousand new cases each year, accounting for more than 40% of the world's total cases [1]. Early detection can significantly improve the survival rate of GC patients (for example, the 5-year survival rate can reach more than 95%) [2], reduce the mortality, and improve the quality of life. However, due to the low early diagnosis rate of GC, most of the patients were in the middle and late stage at the initial diagnosis and had lost the best period of surgical treatment.

The article "Icariin Regulates the hsa_circ_0003159/eIF4A3/bcl-2 Axis to Promote Gastric Cancer Cell Apoptosis" was published in 2022. Journal: Evid Based Complement Alternat Med.

Icariin (ICA) is extracted from Herba Epimedium [3]. As one of the main biologically active compounds from Herba Epimedium, ICA has a variety of pharmacological activities, including anti-inflammatory [4], antiosteoporosis [5, 6], cardiovascular system protection [7], and neuroprotective effects [8]. ICA could enhance the radiotherapy efficacy in the mouse colorectal cancer model [9] and doxorubicin cytotoxicity in drug-resistant osteosarcoma cells [10]. And, ICA can inhibit a variety of tumor cell proliferation and metastasis, effectively inducing tumor cell apoptosis [11]. In GC, ICA increased the proportion of GC cells in the G0/*G*1 phase [12] and inhibited the invasion and migration [13]. However, the molecular mechanism of ICA inhibiting GC is not clear.

CircRNAs are a class of endogenous noncoding RNA molecules with a closed loop structure [14, 15]. It is reported that significantly downregulated circ_0003159 in GC tissues is produced by CACNA2D1 gene [16]. The main mechanism by which circRNAs play a role is through sponging miRNAs or direct interaction with RNA-binding proteins (RBPs) [17–21]. As reported in our published article [22], circ_0003159 inhibits the progression of GC by regulating the miR-223-3p/NLRP3 axis. The eukaryotic initiation factor 4A-3 (eIF4A3), known as an RBP, is a member of the DEAD box family of proteins, and its RNA unwinding activity can unwrap the secondary structure of the mRNA 5′-untranslated region and facilitate the scanning of the 40S ribosomal subunit for the initiation codon. The abnormal structure and function of eIF4A3 can directly affect the transcription and translation of downstream genes [23]. Previous studies showed that circRNA could inhibit the expression of downstream target gene mRNA by binding eIF4A3 [24, 25]. In addition, EIF4A3-binding bcl-2 mRNA was verified with SILAC-based quantitative proteomics [26]. Therefore, we speculate circ_0003159 is involved in GC cell viability and apoptosis by blocking the recruitment of eIF4A3 to bcl-2 mRNA. Our previous studies have reported that ICA regulated circ_0003159/miR-223-3p/NLRP3 axis to promote GC cell pyroptosis [22]. Taken together, it is thus speculated that ICA regulates the hsa_circ_0003159/eIF4A3/bcl-2 axis to promote cell apoptosis of GC cells.

## 2. Materials and Methods

### 2.1. Cell Purchase and Culture

HGC-27 and BGC-803 cell were obtained from BeNa Culture Collection (Beijing, China) and cultured in RPMI-1640 containing 10% FBS (TermoFisher, Wilmington, DE) and penicillin-streptomycin at 37°C in a humidified 5% CO_2_ incubator.

### 2.2. Cell Transfection

The circ_0003159 overexpression plasmid, eIF4A3 overexpression plasmid, and the empty plasmid (vector or NC) were purchased from YRBIO (Changsha, China). eIF4A3 siRNA (si-eIF4A3, 5′-AGACAUGACUAAAGUGGAA-3′) and the negative control sequences were designed and synthesized by GenePharma (Shanghai, China). The GC cells were transfected with the plasmid or siRNA by the Lipofectamine 3000 reagent (Invitrogen, CA, USA). After 24 h later, ICA was added into the GC cell culture and culture together for 48 h.

The article "Icariin Regulates the hsa_circ_0003159/eIF4A3/bcl-2 Axis to Promote Gastric Cancer Cell Apoptosis" was published in 2022. Journal: Evid Based Complement Alternat Med.

### 2.3. Cell Viability Assay

The GC cell viability in this study is tested with the CCK-8 kit (AbMole, USA). In short, CCK-8 reaction solution was added into the treated cell culture and incubated for 4 h, and then the optical density (OD) value (450 nm) was measured to evaluate the cell viability.

### 2.4. RIP Experiment

The RIP assay was performed to determine the endogenous interaction between eIF4A3 and circ_0003159/bcl-2. In brief, BGC-803 and HGC-27 cell lines were lysed in lysis buffer and incubated overnight with magnetic beads conjugated with anti-eIF4A3 antibody on rotation at 4°C. Subsequently, RIP wash buffer was used to wash the bead-antibody complex. RNA was digested with protease K and purified with phenol chloroform. Finally, the immunoprecipitated RNA was extracted and detected by the RT-qPCR assay.

### 2.5. RNA Pull-Down Experiment

The Magnetic RNA-Protein Pull-Down kit was used to detect the interaction between eIF4A3 protein and circ_0003159. HGC-27 and BGC-803 cells were collected and lysed. The biotinylated hsa_circ_0003159 probe was synthesized by Sangon Biotech (Shanghai, China) and incubated with streptavidin agarose beads (Thermo Scientific) for one night at 4°C. The RNA pull-down protein was further analyzed by the western blot assay.

### 2.6. Cell Apoptosis Assay

The Annexin V-PI kit was sued to detect cell apoptosis. The cells were collected, resuspended, and subsequently labeled with Annexin V-FITC and PI. Then, flow cytometry was used to detect cell apoptosis. Finally, the cell apoptosis rate was analyzed by FlowJo software.

### 2.7. qRT-PCR Analysis

Trizol reagent was used to extract total RNA from cells. RNA was used to synthesize cDNA, which was then mixed with SYBR mixture and quantified by real-time PCR. Actin was used as the control. The 2^−ΔΔCT^ method was used to calculate the relative expressions of mRNA. Specific primers for each gene were as follows: bcl-2: forward, 5′-ATCGCCCTGTGGATGACTGAGT-3′ and reverse, 5′-GCCAGGAGAAATCAAACAGAGGC-3'; hsa_circ_0003159: forward, 5'-CCGAACATCTGTCTCCGAAA-3'; reverse, 5'-CTGCTGCGTGCTGATAAGAT-3'; eIF4A3:forward, 5'-CCCTCACCA CAATGACAGCA-3'; reverse, 5'-TGACCCACGCAGGTTaaaca-3'; actin: forward, 5'- CATGTACGTTGCTATCCAGGC -3'; reverse, 5'- CTCCTTAATGTCACGCACGAT -3'.

The article "Icariin Regulates the hsa_circ_0003159/eIF4A3/bcl-2 Axis to Promote Gastric Cancer Cell Apoptosis" was published in 2022. Journal: Evid Based Complement Alternat Med.

### 2.8. Western Blot

HGC-27 and BGC-803 cells were collected and lysed using RIPA Lysis. The BCA Protein Assay Kit (Beyotime Biotechnology, Shanghai, China) was used to measure protein concentration. After quantification, about 30ug protein was separated by SDS-PAGE and then transferred to PVDF membranes. The membrane was incubated with skim milk, then incubated with primary antibodies overnight, and then with the HRP bound secondary antibody for 1 h. The primary antibodies against eIF4A3 (1:200, ab123151), GAPDH (1:1000, ab8245), LaminB1 (1:200, ab65986) and bcl-2 (1:1000, ab117115), and actin (1:1000, ab8226). The protein was observed by enhanced chemiluminescence, and the band intensity was analyzed by the ECL kit.

### 2.9. Statistics

Data were represented as the mean ± SD. The comparisons between the two groups were performed by Student's *t*-test. The comparisons among three or more than three groups were performed by one-way analysis of variance (ANOVA). *P* < 0.05 was considered statistically significant.

## 3. Results

### 3.1. Validation of Interaction between hsa_circ_0003159 and eIF4A3 or eIF4A3 and Bcl-2

To overexpression of circ_0003159 in GC cell, BGC-803 and HGC-27 cell were transfected with the circ_0003159 overexpression plasmid (circ_0003159) and empty plasmid (vector). The nuclear and cytoplasmic proteins were separately extracted and measured, and the western blotting results showed that the ratioof cytoplasmic eIF4A/nuclear eIF4A in the hsa_circ_0003159 overexpression group was higher than that in the Vector group (Figures 1(a)–1(c)). The RIP assay using anti-eIF4A3 showed the higher precipitation of circ_0003159 with the eIF4A3 antibody in GC cells that were transfected with the circ_0003159 overexpression plasmid (Figure 1(d)). RNA pull down further validated the combination relationship between circ_0003159 and eIF4A3 (Figure 1(e)). The RIP assay using anti-eIF4A3 showed the enrichment of bcl-2 mRNA in BGC-803 and HGC-27 cell lines (Figure 1(f)). Moreover, BGC-803 and HGC-27 cells were transfected with si-eIF4A3 followed by actinomycin *D* treatment, and the data showed that the bcl-2 mRNA expression was decreased by actinomycin *D* in a dose-dependent manner in BGC-803 and HGC-27 cell lines, and the bcl-2 mRNA expression was further decreased in the si-eIF4A3 transfection group (Figures 1(g) and 1(h)). The above results show the interaction between circ_0003159 and eIF4A3 protein or eIF4A3 protein and bcl-2 mRNA.

### 3.2. Hsa_circ_0003159 Recruits eIF4A3 to Promote bcl-2 mRNA Degradation

Based on the above investigations, the following study was designed to validate the regulatory pathway axis, hsa_circ_0003159/eIF4A3/bcl-2. HGC-27 and BGC-803 cells were cotransfected with the circ_0003159 overexpression plasmid and si-eIF4A3 or the eIF4A3 overexpression plasmid. The qRT-PCR and western blot data showed that the bcl-2 expressions were downregulated in GC cell by si-eIF4A3 or circ_0003159 overexpression, while it was aggravated by cotransfected with the circ_0003159 overexpression plasmid and si-eIF4A3 (Figures 2(a)–2(c)). On the contrary, the expressions of bcl-2 were upregulated by eIF4A3 overexpression, while it was reversed by cotransfected with circ_0003159 overexpression and eIF4A3 overexpression (Figures 2(d)–2(f)). The RIP assay using anti-bcl-2 showed the lower precipitation of circ_0003159 with the bcl-2 antibody in circ_0003159 overexpressed GC cells (Figure 2(g)). Circ_0003159 overexpression decreased bcl-2 mRNA expression, which was reversed by eIF4A3 overexpression (Figures 2(h) and 2(i)). These results indicate that hsa_circ_0003159 recruits eIF4A3 to inhibit bcl-2 expression.

The article "Icariin Regulates the hsa_circ_0003159/eIF4A3/bcl-2 Axis to Promote Gastric Cancer Cell Apoptosis" was published in 2022. Journal: Evid Based Complement Alternat Med.

### 3.3. Hsa_circ_0003159 Increases GC Cell Apoptosis via eIF4A3/bcl-2

As shown in Figures 3(a) and 3(b), overexpression of circ_0003159 reduced GC cell viability, while eIF4A3 overexpression reversed the effects of circ_0003159 overexpression on the cell viability. The flow cytometry experiment showed that overexpression of circ_0003159 induced GC cell apoptosis, but eIF4A3 overexpression also reversed the induction effects of circ_0003159 overexpression on cell apoptosis (Figures 3(c) and 3(d)). These results suggest that overexpression of eIF4A3 reverses the effect of hsa_circ_0003159 overexpression on GC cell viability and apoptosis.

### 3.4. ICA Regulates the circ_0003159/eIF4A3/bcl-2 Axis to Promote GC Cell Apoptosis

ICA treatment significantly increased circ_0003159 expression but downregulated bcl-2 expression in GC cells (Figures 4(a)–4(d)). Moreover, ICA significantly promoted GC cell apoptosis, and circ_0003159 overexpression aggravated the promotive effect, which was reversed by eIF4A3 overexpression vectors (Figures 4(e) and 4(f)). These findings suggest that ICA regulates hsa_circ_0003159/eIF4A3/bcl-2 axis to promote GC cell apoptosis.

## 4. Discussion

CircRNAs may have an important clinical value in the diagnosis and treatment of GC. It was reported that the downregulated hsa_circ_0003159 in GC [16] is associated with lower overall survival [17]. Further studies found [17] that hsa_circ_0003159 plays a tumor suppressive role in GC. However, its molecular mechanism in GC has not been fully elucidated.

This study firstly showed that the ratio of cytoplasmic eIF4A/nuclear eIF4A in the hsa_circ_0003159 overexpression group was higher than that in the Vector group, and this result was consistent with a previous conclusion [24]. eIF4A3 is a core protein of the EJC and could bind to several spliced mRNAs to affect events primarily in the nucleus [24]. RIP and RNA pull down assays validated the interaction between circ_0003159 and eIF4A3. This is the first study showing the interaction between hsa_circ_0003159 and eIF4A3.

The article "Icariin Regulates the hsa_circ_0003159/eIF4A3/bcl-2 Axis to Promote Gastric Cancer Cell Apoptosis" was published in 2022. Journal: Evid Based Complement Alternat Med.

A previous study indicated that eIF4A3 controls several apoptosis regulators, which are alternatively spliced to produce heterodimers with opposite functions [27]. Consistently, the RIP assay further validated the regulatory relationship between eIF4A3 and bcl-2 mRNA. By gain or loss of the functional experiment, hsa_circ_0003159 was proved to recruit eIF4A3 to inhibit bcl-2 expression. Studies have proved that eIF4A3 regulates tumor cell function and drug resistance by regulating the TNF-*α*/NF-kB signaling pathway [23], whether this signaling pathway was involved ineIF4A3-regulated GC carcinogenesis needs further investigation.

Here, we have demonstrated that circ_0003159 regulates GC cell viability and apoptosis via eIF4A3/bcl-2. Research showed that ICA increases the proportion of GC cells in the G0/G1 phase and significantly inhibited the GC cell invasion and migration [12, 13]. And our previous studies reported ICA regulated hsa_circ_0003159/miR-223-3p/NLRP3 axis to promote GC cell pyroptosis [22]. Other involved important signaling pathways need further investigation.

## 5. Conclusion

This study indicated ICA regulates the hsa_circ_0003159/eIF4A3/bcl-2 axis to promote GC cell apoptosis. This study revealed the molecular target and mechanism of ICA inhibiting gastric cancer and provided a theoretical basis for clinical application of ICA in the treatment of GC.

## Figures and Tables

**Figure 1:** Validation of interaction between hsa_circ_0003159 and eIF4A3 or eIF4A3 and Bcl-2. ((a)–(c)) Western blotting showed the elF4A3 expression in the cytoplasm and nucleus in GC cell lines transfected with circ_0003159 overexpression plasmid (circ_0003159) or empty plasmid (Vector), and the ratio was quantified. (d) RNA immunoprecipitation (RIP) of elF4A3 in GC cell lines that transfected with circ_0003159 or Vector. Circ_0003159 or GAPDH bound to elF4A3 were determined using qRT-PCR. Input of circ_0003159 was normalized to the Vector group. (e) RNA Pull down experimental result indicated the interaction between hsa_circ_0003159 and eIF4A3. (f) Using anti-eIF4A3, RIP experimental result showed the enrichment of bcl-2 in the lysates from GC cell. (g) BGC-803 and (h) HGC-27 cell were transfected with si-eIF4A3 followed by Actinomycin D treatment, and the bcl-2 mRNA expression was quantified by qRT-PCR. ^*∗*^*p* < 0.05 vs. Vector group or siRNA group.

The article "Icariin Regulates the hsa_circ_0003159/eIF4A3/bcl-2 Axis to Promote Gastric Cancer Cell Apoptosis" was published in 2022. Journal: Evid Based Complement Alternat Med.

**Figure 2:** Hsa_circ_0003159 inhibit bcl-2 expression by recruiting eIF4A3 protein. (a) qRT-PCR detected the bcl-2 mRNA expression in GC cell transfected with circ_0003159 overexpression vector and/or si-eIF4A3. ((b)-(c)) Western blotting detected showed the bcl-2 protein expression in GC cell transfected with circ_0003159 overexpression vector and/or si-eIF4A3. (d) qRT-PCR detected the bcl-2 mRNA expression in GC cell transfected with circ_0003159 and/or eIF4A3 overexpression vector. ((e)-(f)) Western blotting detected showed the bcl-2 protein expression in GC cell transfected with circ_0003159 and/or eIF4A3 overexpression vector. (g) RIP of bcl-2 in GC cell after transfection with circ_0003159 or Vector. Circ_0003159 and GAPDH bound to bcl-2 were determined using qRT-PCR. Input of circ_0003159 was normalized to the Vector group. (h) BGC-803 and (i) HGC-27 cell were transfected with circ_0003159 and/or eIF4A3 overexpression vector, followed by Actinomycin D treatment, and the bcl-2 mRNA expression was quantified by qRT-PCR. ^*∗*^*p* < 0.05 vs. Vector + siRNA/NC or Vector group. ^#^*p* < 0.05 vs. circ_0003159 + si-eIF4A3/NC or circ_0003159 group.

**Figure 3:** Hsa_circ_0003159 regulates eIF4A3/bcl-2 to reduce GC cell viability and increase cell apoptosis. The (a) BGC-803 and (b) HGC-27 cell viability were detected by CCK8 assay. Flow cytometry experiment showed the BGC-803 (c) and HGC-27 (d) cell apoptosis. ^*∗*^*p* < 0.05 vs. Vector. ^#^*p* < 0.05 vs. circ_0003159.

**Figure 4:** ICA regulates hsa_circ_0003159/eIF4A3/bcl-2 axis to promote GC cell apoptosis. (a) qRT-PCR data showed ICA significantly upregulated the expression of hsa_circ_0003159. (b) qRT-PCR assay showed ICA significantly downregulated the bcl-2 mRNA expression GC cells. ((c)-(d)) Western blotting assay showed that ICA significantly downregulated the bcl-2 protein expression in GC cell. ((e)-(f)) Flow cytometry experiment showed GC cell apoptosis. ^*∗*^*p* < 0.05 vs. Vehicle or ICA + vector. ^&^*p* < 0.05 vs. Control. ^#^*p* < 0.05 vs. ICA + circ_0003159.

## Data Availability

The data used and analyzed during the current study are available from the first author and corresponding author on reasonable request.
